# Accumulation of Phosphorylated β-Catenin Enhances ROS-Induced Cell Death in Presenilin-Deficient Cells

**DOI:** 10.1371/journal.pone.0004172

**Published:** 2009-01-12

**Authors:** Jung H. Boo, Hyundong Song, Ji E. Kim, David E. Kang, Inhee Mook-Jung

**Affiliations:** 1 Interdisciplinary Program in Brain Science, School of Biological Sciences, Seoul National University College of Medicine, Seoul, Korea; 2 Department of Biochemistry and Biomedical Sciences, Seoul National University College of Medicine, Seoul, Korea; 3 Department of Neurosciences, University of California San Diego, La Jolla, California, United States of America; Ordway Research Institute, United States of America

## Abstract

Presenilin (PS) is involved in many cellular events under physiological and pathological conditions. Previous reports have revealed that PS deficiency results in hyperproliferation and resistance to apoptotic cell death. In the present study, we investigated the effects of PS on β-catenin and cell mortality during serum deprivation. Under these conditions, PS1/PS2 double-knockout MEFs showed aberrant accumulation of phospho-β-catenin, higher ROS generation, and notable cell death. Inhibition of β-catenin phosphorylation by LiCl reversed ROS generation and cell death in PS deficient cells. In addition, the K19/49R mutant form of β-catenin, which undergoes normal phosphorylation but not ubiquitination, induced cytotoxicity, while the phosphorylation deficient S37A β-catenin mutant failed to induce cytotoxicity. These results indicate that aberrant accumulation of phospho-β-catenin underlies ROS-mediated cell death in the absence of PS. We propose that the regulation of β-catenin is useful for identifying therapeutic targets of hyperproliferative diseases and other degenerative conditions.

## Introduction

β-catenin is a multifunctional protein that forms an adhesion complex with E-cadherin, α-catenin, and actin; it also plays a central role in Wnt signaling through its nuclear translocation and association with T-cell factor (TCF) and lymphoid enhancer factor (LEF) [1], [2]. Cytosolic β-catenin is tightly regulated by interactions with several proteins, such as adenomatous polyposis coli (APC), glycogen synthase kinase-3β (GSK-3β), and axin [3], [4]. β-catenin is sequentially phosphorylated at serine 45 by casein kinase-1 (CK-1) and at threonine 41, serine 37, and serine 33 by GSK-3β. Phosphorylated β-catenin is recognized by β-transducin repeat-containing protein (β-TrCP) E3 ligase, which targets it for degradation by ubiquitin-proteasomal machinery [5]–[7].

Presenilin (PS) is a multipass membrane protein that regulates many physiological and pathological processes. Mutations in two PS genes, PS1 and PS2, cause familial Alzheimer disease (FAD) and elevate levels of the longer form of amyloid β-peptide (Aβ), which is derived from amyloid precursor protein (APP) [8], [9]. PS is the catalytic subunit of the γ-secretase complex that cleaves many type 1 membrane proteins. Besides its activity in the γ-secretase complex, PS has effects on various intracellular activities, such as Wnt/β-catenin signaling, phosphatidylinositol 3-kinase/Akt and MEK/ERK signaling, calcium homeostasis, and apoptosis [10]–[14]. PS1-null mice are embryonic lethal and exhibit skeletal and central nervous system (CNS) defects [15]. Studies of mouse embryonic fibroblasts (MEFs) from PS1-null mice and skin of adult PS1 conditional knockout mice, however, show that PS1 deficiency elicits tumor-like phenomena at least in part through stabilization of β-catenin and epidermal growth factor receptor (EGFR) [10], [16], [17]. In addition, PS deficiency and inhibition of γ-secretase activity cause resistance to apoptotic stimuli [14], [18].

In the present study, we identified a novel function of phosphorylated β-catenin in the absence of PS. Phosphorylated β-catenin accumulated abnormally in PS-deficient MEFs under conditions of serum deprivation, provoking reactive oxygen species (ROS) generation and ROS-induced cell death.

## Results

### PS dKO MEFs are vulnerable to serum deprivation-induced cell death

Although we confirmed protein expression of PS1 and nicastrin in crude extracts of PS WT and human PS1-rescued PS dKO (hPS1) MEFs, PS was not detected in PS dKO MEFs, as previously reported [19]. Immature form of nicastrin was detected in PS dKO cells as expected. Exogenous human PS1, however, recovered the PS1-CTF band and maturation of nicastrin (Figure 1A). To examine the role of PS in cell survival, conditions of serum deprivation were applied to each cell type. By LDH release assay, PS dKO MEFs were more vulnerable to serum deprivation than PS WT cells (p<0.001, Figure 1B). Restoration of hPS1 in PS dKO MEF decreased this vulnerability and restored the rate of cell death to PS WT levels (p<0.001, Figure 1B).

**Figure 1:** PS dKO MEFs are vulnerable to serum deprivation-induced cell death. (A) Western blot analysis of nicastrin and PS1 showing that PS dKO MEFs prevent nicastrin maturation. hPS1 MEFs were rescued PS1 and nicastrin maturation. Calnexin served as a loading control for membrane fractions. Filled and blank arrows indicate mature and immature nicastrin, respectively. Filled and blank arrowheads indicate full-length PS1 and PS1-CTF, respectively. (B) LDH release assay showing that PS dKO MEFs are injured by serum deprivation-induced stress. All MEFs were incubated DMEM media without serum for 36 hr. The graph represents (%) of positive control. Data are means±SEM values of three independent experiments. * represents significant differences from PS WT MEFs. ***P<0.001. # represents significant differences from PS dKO MEFs. ###P<0.001.

### Serum deprivation accentuates ROS generation in PS dKO MEFs

To determine the mechanism that underlies serum deprivation-induced cell death in PS dKO MEFs, we examined ROS generation in these MEFs by fluorescence microscopy using the DCFDA fluorophore. After 36 hr in DMEM, PS dKO MEFs generated high levels of ROS, as evidenced by damaged morphology with DCFDA staining (Figure 2A). Unlike PS dKO MEFs, PS WT and hPS1 MEFs had healthier cell morphologies, exhibiting lower DCFDA signals (Figure 2A). We also assessed the effects of trolox, a water-soluble derivative of vitamin E, as an antioxidant and LiCl, a widely used GSK-3 inhibitor, on stress from serum deprivation. Trolox and LiCl treatment protected PS dKO MEFs against serum deprivation-induced cell death (p<0.001, Figure 2B) and inhibited ROS generation (Figure 2A).

**Figure 2:** ROS-mediated serum deprivation-induced cell death in PS dKO MEFs. (A) ROS generation of MEFs was detected using the DCFDA fluorophore. All MEFs were incubated in DMEM w/wo 200 µM trolox or 10 mM LiCl for 36 hr. PS dKO MEFs showed higher signal intensities, but hPS1-rescued MEFs and trolox- or LiCl -treated PS dKO MEFs had lower signals. The white bar represents 50 µm. (B) PS dKO MEFs were incubated in the presence or absence of 200 µM trolox or 10 mM LiCl in DMEM for 36 hr. LDH release assay showed that both trolox and LiCl efficiently protected against serum deprivation-induced cell death. The graph represents (%) of positive control. Data are means±SEM values of three independent experiments. * represents significant differences from untreated PS dKO MEFs. ***P<0.001.

### Phospho-β-catenin accumulates in PS dKO MEFs under serum deprivation

We examined β-catenin protein levels in PS dKO MEFs because PS interacts with β-catenin [20]. By Western blot, we observed higher levels of β-catenin in PS dKO MEFs, but β-catenin levels in hPS1 MEFs and PS WT MEFs were comparable in basal condition (Figure 3A). Based on our results that LiCl treatment protected PS dKO MEFs against serum deprivation induced-ROS generation and cell death (Figure 2A and 2B, respectively), we investigated the effect of GSK-3β on β-catenin phosphorylation. By immunofluorescence using a specific antibody for phospho-β-catenin (S33, S37, and T41), we detected robust phospho-β-catenin signals in PS dKO MEFs under conditions of serum deprivation, but PS WT MEFs in either growth or serum-deprived media and PS dKO MEFs in growth media showed little fluorescence (Figure 3B). In PS dKO MEFs, GSK-3β inhibition with LiCl reduced phospho-β-catenin levels (S33, S37, T41), but trolox did not (Figure 3C), as confirmed by Western blot (Figure 3D).

**Figure 3:** Phospho-β-catenin was accumulated in PS dKO MEFs under serum deprivation conditions. (A) β-catenin was accumulated in PS dKO MEFs, not in PS WT under normal and serum deprivation conditions. β-actin served as a loading control. (B) PS WT and PS dKO MEFs were incubated in growth media or DMEM for 30 hr, followed by immunofluorescent staining. PS dKO MEFs in DMEM labeled more brightly against anti-phospho-β-catenin (S33, 37, T41) antibody. The white bar represents 200 µm. (C) PS dKO MEFs were incubated w/wo 10 mM LiCl or 200 µM trolox in DMEM for 30 hr and labeled with phospho-β-catenin (S33, 37, T41)-specific antibody (Red). Many cells contained phosphorylated forms of β-catenin in DMEM- and trolox-treated PS dKO MEFs by fluorescence microscopy. But, LiCl-treated PS dKO MEFs stained weakly. DAPI staining was used to visualize cell nuclei (Blue). The white bar represents 200 µm. (D) Western blot analysis showed that LiCl effectively decreased phosphorylation of β-catenin at the S33, 37, and T41 sites without altering total β-catenin or β-actin levels. However, trolox-treated cells showed similar levels of phospho-β-catenin compared with DMEM alone.

### Accumulation of phospho-β-catenin induces cytotoxicity in H4 neuroglioma cells

To examine whether accumulated phospho-β-catenin affects cell viability, we introduced several β-catenin constructs into H4 neuroglioma cells. After transient transfection with each construct, we measured protein expression from these constructs in H4 cells. To induce phospho-β-catenin accumulation, the K19/49R mutant construct was transfected, because this mutant fails to undergo ubiquitination and degradation due to their mutated ubiquitination site [7]. By Western blot, levels of the phosphorylated form of β-catenin (on residues 33, 37, and 41) were high in K19/49R β-catenin mutant transfectants (Figure 4A), suggesting that phospho-β-catenin accumulated in the cells. In contrast, the S37A β-catenin mutant induced the highest levels of total β-catenin but showed low reactivity by immunoblotting with anti-phospho-β-catenin (Figure 4A). Endogenous β-catenin and β-actin in each transfectant cell type were expressed similarly. Using these constructs, we performed the LDH release assay to measure cell viability under conditions of serum deprivation. K19/49R β-catenin mutant-transfected H4 cells had increased rates of cell death compared with WT β-catenin-transfected cells (p<0.005, Figure 4B); S37A β-catenin-transfected H4 cells, however, had greater viability compared with WT β-catenin transfectants (p<0.05, Figure 4B). To determine the effects of phospho-β-catenin on ROS generation, we stained H4 cells with DCFDA. Similar to the results of the LDH release assay, most K19/49R β-catenin transfectants were brightly stained, although only few cells remained (Figure 4C). WT β-catenin and S37A β-catenin transfectants did not stain as intensely as the K19/49R transfectants (Figure 4C), suggesting that accumulation of phospho-β-catenin induces ROS generation.

**Figure 4:** Accumulation of phospho-β-catenin induces cytotoxicity in H4 neuroglioma cells. (A) H4 cells were transiently transfected with EYFP vector, WT, and mutant β-catenin constructs in DMEM for 16 hr. K19/49R β-catenin-transfected cells showed higher immunoreactivity against anti-phospho-β-catenin (S33, 37, T41) without affecting endogenous β-catenin and β-actin levels. Filled and blank arrows indicate exogenous β-catenin-EYFP fusion protein and endogenous β-catenin, respectively. Arrowhead indicates nonspecific bands. (B) LDH release assay showed that K19/49R β-catenin induced cytotoxicity in the transfectants. The graph represents (%) of positive control. Data are means±SEM values of three independent experiments. * represents significant differences from EYFP vector-transfected H4 cells. *P<0.05, **P<0.01, ***P<0.001. # represents significant differences from WT β-catenin-EYFP-transfected H4 cells. ###P<0.001. (C) DCFDA staining showing ROS generation of mock and β-catenin-transfected H4 cells. Although fewer cells remained among K19/49R β-catenin tranfectants, the DCFDA signal was much higher than in other transfectants. The white bar represents 200 µm.

## Discussion

PS performs many functions in such physiological and pathological processes as development, calcium signaling, apoptosis, and Alzheimer disease. Previous studies demonstrated that β-catenin accumulation occurs in the absence of PS, which is accompanied by increased proliferation [16], [17]; these results were recapitulated in our experiments in which PS dKO MEFs experienced an accumulation in β-catenin (Figure 3A) and increased proliferation (data not shown) in normal growth media. In contrast, several reports have shown that β-catenin suppresses growth and induces cytotoxicity [21]–[23]. Here, we examined cell mortality and β-catenin expression under conditions of serum deprivation in the absence of PS. Because PS dKO MEFs died easily on removal of serum compared with PS WT MEFs, we determined whether PS was associated with this phenomenon using hPS1-supplied MEFs. Reconstitution of human PS1 in PS dKO MEFs reversed the vulnerability to serum deprivation-induced cell death, suggesting that PS1 is protective under such circumstances.

To identify the underlying mechanism of these phenomena, intracellular ROS levels were measured, because ROS are formed during serum deprivation-induced cell death [24], although there has been no report that links between β-catenin and ROS generation. Many cells were stained brightly with DCFDA in PS dKO MEFs during serum deprivation, but PS-containing MEFs and LiCl- and trolox-treated PS dKO MEFs experienced reduced fluorescent intensity and cell death. When PS dKO MEFs were deprived of serum, they accumulated more phospho-β-catenin, generated more ROS, and died at higher rates than PS WT MEFs or hPS1 MEFs. Treatment with the antioxidant trolox inhibited ROS generation and serum deprivation-induced cell death in PS dKO MEFs (Figure 2A & B), but it could not block phospho-β-catenin levels (Figure 3C & D). Treatment with LiCl, a potent inhibitor that blocks the phosphorylation of β-catenin by GSK-3β, reduced phospho-β-catenin levels, ROS generation, and serum deprivation-induced cell death in PS dKO MEFs (Figures 2A & B and Figures 3C & D). These results suggest that accumulation of phospho-β-catenin causes the generation of ROS and cell death in serum-deprived PS dKO MEFs. To assess the cytotoxic effect of GSK-3β-induced phospho-β-catenin, we transiently transfected H4 neuroglioma cells with wild-type and mutant β-catenin constructs. Because β-catenin undergoes sequential processing, including phosphorylation, ubiquitination, and degradation, we designed an experiment with various β-catenin mutants, in which we substituted serine for alanine at position 37. This mutation inhibited GSK-3β-mediated phosphorylation of β-catenin, curtailing subsequent ubiquitination and proteosomal degradation. Substitution of lysine with arginine at positions 19 and 49 inhibited ubiquitination of β-catenin and degradation as well. Western blot analysis with anti-phospho-β-catenin (S33, 37, T41) demonstrated that the K19/49R β-catenin mutant had the highest immunoreactivity, as expected. The S37A β-catenin mutant was robustly detected by an anti-β-catenin antibody that recognized the total protein but had low immunoreactivity against the GSK-3β-mediated phospho-β-catenin antibody. This mutant was well labeled by anti-phospho-β-catenin (T41, S45), as expected (data not shown). In contrast, because exogenous WT β-catenin also was regulated by endogenous machinery, little exogenous WT β-catenin remained in the β-catenin mutants. In the LDH release assay, K19/49R β-catenin mutant-transfected H4 cells had higher rates of cell death and ROS generation than transfectants of other mutants. S37A β-catenin-transfected H4 cells experienced less death and ROS generation than wild-type β-catenin transfectants, despite higher total levels of β-catenin in S37A β-catenin mutant transfectants than in K19/49R β-catenin transfectants and wild-type cells (Figure 4). These results imply that increases in β-catenin are not essential in generating ROS or inducing cell death under conditions of serum deprivation. Only accumulation of phospho-β-catenin is responsible for ROS generation and the ensuing cell death. This is the first report that demonstrates that accumulation of phospho-β-catenin generates ROS and leads to cell death in a PS-dependent manner. It is to be clarified why phospho-β-catenin is more toxic. It maybe phosphorylation changes the conformation of β-catenin such that it may interact with proteins in a different way or inhibits the E3 ligase machinery. Or, it may not be the phosphorylation per se, but the activity of GSK-3, β-TrCP E3 ligase, or proteasome [25]–[27]. We checked whether γ-secretase inhibitor can mimic the increased vulnerability to serum withdrawal using PS expressing cells. Since γ-secretase inhibitor did not affect vulnerability of the cells, we can rule out intramembrane proteolysis, and β-catenin is not regulated by γ-secretase inhibitor under serum deprivation condition. One other point is why serum deprivation preferentially increases β-catenin phosphorylation in the absence of PS. Under normal basal conditions, we previously showed that PS facilitates β-catenin phosphorylation via a scaffolding mechanism (bringing β-catenin and GSK-3 in complex with PS). At the same time, generalized GSK-3 activity (as detected by phospho-GSK3) is increased in PS dKO cells. Serum withdrawal should further enhance general GSK-3 activity in all cells because of lack of growth factor, etc. and loss of PI3K/Akt signaling [28], [29]. But perhaps under conditions of prolonged serum withdrawal (36 hrs), GSK-3 activity, localization, etc may be altered (i.e. directed at tau for example) such that PS1 still sequesters β-catenin but cannot bring together GSK-3. If so, then the loss of PS may indirectly promote GSK-3 mediated phosphorylation of β-catenin by neither sequestering β-catenin nor GSK-3. These points are needed to be clarified by further study.

Taken together, β-catenin facilitates cell proliferation under normal growth conditions, but when serum is limited, phosphorylated β-catenin accumulates in the absence of PS and induces ROS generation and cell death.

## Materials and Methods

### Cell culture and transfection

Wild-type (PS+/+) MEFs (PS WT MEFs), PS double knockout (PS−/−; ie, doubly deficient for PS1 and PS2) MEFs (PS dKO MEFs) (a kind gift from Dr. Bart De Strooper, Katholieke Universiteit Leuven, Leuven, Belgium), and PS−/− MEFs that stably expressed human wild-type PS1 (hPS1) (hPS1 MEFs) were maintained according to previous reports [13], [30], [31]. Briefly, the human neuroglioma cell line H4 and all MEFs were maintained in Dulbecco's modified Eagle's medium (DMEM; HyClone, Salt Lake City, Utah) supplemented with 10% fetal bovine serum (FBS; HyClone) and 0.1 mg/ml penicillin and streptomycin (Sigma, St Louis, MO) at 37°C in a 5% CO_2_ incubator. Transient transfection was performed using LipofectAMINE LTX (Invitrogen, Carlsbad, CA) according to the instructions provided by the manufacturer.

### Plasmids and antibodies

Wild-type β-catenin (a kind gift form Dr. CY Choi, Sungkyunkwan University, Korea), and each mutant (S37A, S45A, or K19/49R) in mock and EYFP vectors were transfected into H4 cells. The following antibodies were used: mouse monoclonal anti-β-catenin (Transduction Laboratories, BD Biosciences, San Jose, CA); rabbit polyclonal anti-phospho-β-catenin (Ser33/37/Thr41), rabbit polyclonal anti-phospho-β-catenin (Thr41/Ser45), and rabbit polyclonal anti-calnexin (Cell Signaling, Beverly, MA); mouse monoclonal anti-nicastrin, and mouse monoclonal anti-PS1 loop (Chemicon, Temecula, CA); and mouse monoclonal anti-β-actin (Sigma).

### Cell viability assay

Dead and membrane-ruptured cells were quantitatively measured by lactate dehydrogenase (LDH) release. Aliquots (50 µl) of cell culture medium were mixed with 0.42 mM β-NADH in potassium phosphate buffer, pH 7.4 (125 µl; sigma) and 20 mM sodium pyruvate (25 µl; Sigma) in a microplate. After being mixed with sodium pyruvate, the samples were measured immediately 7 times at 340 nm for 5 min. Kinetic measurements were monitored using a microplate spectrophotometer (PowerWave XS; BIO-TEK instruments Inc., Winooski, VT). We used 0.5% Triton X-100-treated samples as positive controls.

### Western blot analysis

Harvested cell pellets were resuspended in RIPA buffer (150 mM NaCl, 1% Nonidet P-40, 0.5% deoxycholic acid, 0.1% SDS, and 50 mM Tris-HCl, pH 7.4) containing protease inhibitors (Sigma) and incubated on ice for 20 min. After centrifugation at 15,000 *g* for 20 min, the supernatant was collected. Crude membrane fractions of the cultured cells were prepared according to previous reports, with minor modifications [32], [33]. Protein concentrations were determined by BCA assay (Sigma), and equal amounts of protein were loaded on appropriate gels. The separated samples were transferred to a PVDF membrane and incubated with antibodies against the target proteins. Protein bands were visualized by enhanced chemiluminescence (ECL; Amersham Pharmacia Biotech, Buckinghamshire, England) using a bioimaging analyzer (LAS-3000; Fuji, Tokyo, Japan).

### ROS measurement

Levels of hydrogen peroxide were determined using dichlorofluorescein diacetate (DCFDA; Invitrogen, Carlsbad, CA). Treated cells were incubated with 10 µM DCFDA for 30 min and washed with PBS. Fluorescent signals were captured using a fluorescence microscope (Olympus, Tokyo, Japan).

### Immunofluorescence

Treated cells were fixed with 2% paraformaldehyde (PFA) for 10 min and washed with PBS. Fixed cells were permeabilized with PBST buffer (0.5% Triton X-100 in PBS) and incubated with blocking solution (2% goat serum and 2% horse serum in PBST) for 1 hr. Cells were incubated with primary antibodies in blocking solution overnight at 4°C. Labeled cells were washed with PBST and relabeled with Cy-3-conjugated secondary antibody. After cells were counterstained with DAPI (Sigma), fluorescent signals were visualized by fluorescence microscopy (Olympus).

### Statistical analysis

All data were expressed as mean±SEM. Significant differences were calculated using one-way ANOVA with Tukey's post-test. A *P* value of less than 0.05 denoted a statistically significant difference.

## References

[1] Aberle H, Schwartz H, Kemler R (1996). Cadherin-catenin complex: protein interactions and their implications for cadherin function.. J Cell Biochem.

[2] Hsu SC, Galceran J, Grosschedl R (1998). Modulation of transcriptional regulation by LEF-1 in response to Wnt-1 signaling and association with beta-catenin.. Mol Cell Biol.

[3] Munemitsu S, Albert I, Souza B, Rubinfeld B, Polakis P (1995). Regulation of intracellular beta-catenin levels by the adenomatous polyposis coli (APC) tumor-suppressor protein.. Proc Natl Acad Sci U S A.

[4] Ikeda S, Kishida S, Yamamoto H, Murai H, Koyama S (1998). Axin, a negative regulator of the Wnt signaling pathway, forms a complex with GSK-3beta and beta-catenin and promotes GSK-3beta-dependent phosphorylation of beta-catenin.. EMBO J.

[5] Liu C, Li Y, Semenov M, Han C, Baeg GH (2002). Control of beta-catenin phosphorylation/degradation by a dual-kinase mechanism.. Cell.

[6] Liu C, Kato Y, Zhang Z, Do VM, Yankner BA (1999). beta-Trcp couples beta-catenin phosphorylation-degradation and regulates Xenopus axis formation.. Proc Natl Acad Sci U S A.

[7] Aberle H, Bauer A, Stappert J, Kispert A, Kemler R (1997). beta-catenin is a target for the ubiquitin-proteasome pathway.. EMBO J.

[8] Sherrington R, Rogaev EI, Liang Y, Rogaeva EA, Levesque G (1995). Cloning of a gene bearing missense mutations in early-onset familial Alzheimer's disease.. Nature.

[9] Hardy J (1997). Amyloid, the presenilins and Alzheimer's disease.. Trends Neurosci.

[10] Soriano S, Kang DE, Fu M, Pestell R, Chevallier N (2001). Presenilin 1 negatively regulates beta-catenin/T cell factor/lymphoid enhancer factor-1 signaling independently of beta-amyloid precursor protein and notch processing.. J Cell Biol.

[11] Pack-Chung E, Meyers MB, Pettingell WP, Moir RD, Brownawell AM (2000). Presenilin 2 interacts with sorcin, a modulator of the ryanodine receptor.. J Biol Chem.

[12] Zhang Z, Hartmann H, Do VM, Abramowski D, Sturchler-Pierrat C (1998). Destabilization of beta-catenin by mutations in presenilin-1 potentiates neuronal apoptosis.. Nature.

[13] Kang DE, Yoon IS, Repetto E, Busse T, Yermian N (2005). Presenilins mediate phosphatidylinositol 3-kinase/AKT and ERK activation via select signaling receptors. Selectivity of PS2 in platelet-derived growth factor signaling.. J Biol Chem.

[14] Alves da Costa C, Sunyach C, Pardossi-Piquard R, Sevalle J, Vincent B (2006). Presenilin-dependent gamma-secretase-mediated control of p53-associated cell death in Alzheimer's disease.. J Neurosci.

[15] Shen J, Bronson RT, Chen DF, Xia W, Selkoe DJ (1997). Skeletal and CNS defects in Presenilin-1-deficient mice.. Cell.

[16] Repetto E, Yoon IS, Zheng H, Kang DE (2007). Presenilin 1 regulates epidermal growth factor receptor turnover and signaling in the endosomal-lysosomal pathway.. J Biol Chem.

[17] Kang DE, Soriano S, Xia X, Eberhart CG, De Strooper B (2002). Presenilin couples the paired phosphorylation of beta-catenin independent of axin: implications for beta-catenin activation in tumorigenesis.. Cell.

[18] Arumugam TV, Chan SL, Jo DG, Yilmaz G, Tang SC (2006). Gamma secretase-mediated Notch signaling worsens brain damage and functional outcome in ischemic stroke.. Nat Med.

[19] Leem JY, Vijayan S, Han P, Cai D, Machura M (2002). Presenilin 1 is required for maturation and cell surface accumulation of nicastrin.. J Biol Chem.

[20] Yu G, Chen F, Levesque G, Nishimura M, Zhang DM (1998). The presenilin 1 protein is a component of a high molecular weight intracellular complex that contains beta-catenin.. J Biol Chem.

[21] Damalas A, Ben-Ze'ev A, Simcha I, Shtutman M, Leal JF (1999). Excess beta-catenin promotes accumulation of transcriptionally active p53.. EMBO J.

[22] Usami N, Sekido Y, Maeda O, Yamamoto K, Minna JD (2003). Beta-catenin inhibits cell growth of a malignant mesothelioma cell line, NCI-H28, with a 3p21.3 homozygous deletion.. Oncogene.

[23] Kim K, Pang KM, Evans M, Hay ED (2000). Overexpression of beta-catenin induces apoptosis independent of its transactivation function with LEF-1 or the involvement of major G1 cell cycle regulators.. Mol Biol Cell.

[24] Pandey S, Lopez C, Jammu A (2003). Oxidative stress and activation of proteasome protease during serum deprivation-induced apoptosis in rat hepatoma cells; inhibition of cell death by melatonin.. Apoptosis.

[25] Pap M, Cooper GM (1998). Role of glycogen synthase kinase-3 in the phosphatidylinositol 3-Kinase/Akt cell survival pathway.. J Biol Chem.

[26] Fuchs SY, Spiegelman VS, Kumar KG (2004). The many faces of beta-TrCP E3 ubiquitin ligases: reflections in the magic mirror of cancer.. Oncogene.

[27] Drexler HC (1997). Activation of the cell death program by inhibition of proteasome function.. Proc Natl Acad Sci U S A.

[28] Brunet A, Bonni A, Zigmond MJ, Lin MZ, Juo P (1999). Akt promotes cell survival by phosphorylating and inhibiting a Forkhead transcription factor.. Cell.

[29] Gerber HP, McMurtrey A, Kowalski J, Yan M, Keyt BA (1998). Vascular endothelial growth factor regulates endothelial cell survival through the phosphatidylinositol 3′-kinase/Akt signal transduction pathway. Requirement for Flk-1/KDR activation.. J Biol Chem.

[30] Herreman A, Hartmann D, Annaert W, Saftig P, Craessaerts K (1999). Presenilin 2 deficiency causes a mild pulmonary phenotype and no changes in amyloid precursor protein processing but enhances the embryonic lethal phenotype of presenilin 1 deficiency.. Proc Natl Acad Sci U S A.

[31] Herreman A, Van Gassen G, Bentahir M, Nyabi O, Craessaerts K (2003). gamma-Secretase activity requires the presenilin-dependent trafficking of nicastrin through the Golgi apparatus but not its complex glycosylation.. J Cell Sci.

[32] Kim SK, Park HJ, Hong HS, Baik EJ, Jung MW (2006). ERK1/2 is an endogenous negative regulator of the gamma-secretase activity.. FASEB J.

[33] Sastre M, Steiner H, Fuchs K, Capell A, Multhaup G (2001). Presenilin-dependent gamma-secretase processing of beta-amyloid precursor protein at a site corresponding to the S3 cleavage of Notch.. EMBO Rep.

